The article "IgG4-Related Disease without Overexpression of IgG4: Pathogenesis Implications" was published in 2012. Journal: Case Rep Rheumatol.

# IgG4-Related Disease without Overexpression of IgG4: Pathogenesis Implications

**DOI:** 10.1155/2012/754935

**Published:** 2012-08-05

**Authors:** Naoshi Nishina, Yuko Kaneko, Masataka Kuwana, Hironari Hanaoka, Hideto Kameda, Shuji Mikami, Tsutomu Takeuchi

**Affiliations:** ^1^Division of Rheumatology, Department of Internal Medicine, School of Medicine, Keio University, 35 Shinanomachi Shinjuku-ku, Tokyo 160-8582, Japan; ^2^Division of Diagnostic Pathology, Keio University Hospital, Tokyo 160-8582, Japan

## Abstract

IgG4-related disease is a new disease group that affects multiple organs. It is characterized by high serum IgG4 and abundant infiltration of IgG4-bearing plasma cells in the affected organ. Here, we describe an intriguing case that suggested that IgG4-related disease might present without IgG4 overexpression or infiltration, at least during a relapse. A 47-year-old man had been diagnosed with systemic lupus erythematosus 15 years. He was admitted due to a pituitary mass, systemic lymphadenopathy, and multiple nodules in the lungs and kidneys. The serum IgG4 level was normal and histopathological examination of the pituitary mass showed abundant lymphocyte and plasma cell infiltration with very few IgG4-positive cells. When we examined specimens preserved from 15 years ago, we found high serum IgG4 levels and IgG4-bearing plasma cell infiltration. This resulted in a diagnosis of IgG4-related disease, and we considered the current episode to be a relapse without IgG4 overexpression. This case indicated that, to clarify the pathogenesis of IgG4-related disease, current cases should repeat specimen evaluations over the course of IgG4-related disease to define diagnostic markers.

## 1. Introduction

IgG4-related disease, first described in 2001 [1], is a new disease group that affects multiple organs. It is characterized by high serum IgG4 and infiltration of the affected organ with lymphoplasmacytes, IgG4-bearing plasma cells, and fibrosis [2–4]. Because high serum IgG4 and abundant infiltration of IgG4-bearing plasma cells are prominent characteristics, it was suggested that these findings could define the diagnosis of IgG4-related disease [5]. However, the pathogenesis of IgG4 overexpression remains unclear [6], and it is unknown whether IgG4 is related to the cause of the disease. 

Here, we described a case of IgG4-related disease that had been exacerbated after 15 years of remission. At the time of the relapse, the patient exhibited several masses in various organs, including pituitary, lung, kidney, and lymph nodes. However, the serum IgG4 level was within normal limits. A histopathological examination of pituitary gland and lung masses showed infiltration of numerous plasma cells, but very few IgG4-bearing cells. This intriguing finding indicated that IgG4-related disease could present without abundant IgG4-bearing plasma cell infiltration, at least at the time of a relapse.

The article "IgG4-Related Disease without Overexpression of IgG4: Pathogenesis Implications" was published in 2012. Journal: Case Rep Rheumatol.

## 2. Case Presentation

In 2010, a 47-year-old Japanese man was admitted to Keio University Hospital due to a vision abnormality.

In 1994, he had visited our hospital with lymphadenopathy. At that time, he had high serum IgG (6098 mg/dL), and a lymph node specimen from the left inguinal area revealed nonspecific lymphoid hyperplasia, which did not define a diagnosis. In 1995, the suspected diagnosis was systemic lupus erythematosus (SLE), based on observations of polyarthritis, low white blood cell count (1600/*μ*L), positivity for antinuclear antibody, and slightly elevated anti-DNA antibody (12.2 IU/mL by radioimmunoassay; normal range <6 IU/mL). He was treated with 20 mg daily prednisolone (PSL) and the symptoms disappeared rapidly. Subsequently, the PSL was gradually tapered down. From 2008, he had been taking 2 mg daily PSL and remained in stable condition until he experienced abnormal vision in 2010. 

In the 2010 admission, a physical examination showed multiple swollen lymph nodes (1.5 cm maximum diameter) in the neck and inguinal area. A visual field examination revealed bilateral hemianopsia. Laboratory blood tests showed normal results for the blood count, serum electrolytes, serum creatinine, liver enzymes, and lactate dehydrogenase. The C-reactive protein level was slightly elevated to 0.86 mg/dL. The total serum IgG was 3189 mg/dL, with 1550 mg/dL IgG1 (normal range, 320–748), 1100 mg/dL IgG2 (normal range, 208–754), 444 mg/dL IgG3 (normal range, 6.6–88.3), and 94.9 mg/dL IgG4 (normal range, 4.8–105). Magnetic resonance imaging (MRI) of the head revealed a pituitary mass of 30 mm (Figure 1(a)), which was considered the cause of bilateral hemianopsia. A computed tomography (CT) scan showed nodules in both lungs and a lesion in the left kidney that was devoid of contrast enhancement (Figures 1(b) and 1(c)). ^67^Gallium scintigraphy showed abnormal accumulation in the pituitary gland, both sides of the neck, lungs, kidneys, and the right inguinal area (Figure 1(d)). Biopsies were taken of the pituitary and lung (transbronchial). Both showed similar pathological findings, including mild fibrosis with abundant infiltration of plasma cells and lymphocytes. Nevertheless, immunohistochemical staining for IgG4 was positive for only about 10% of all IgG-positive plasma cells (Figures 2(a) and 2(b)). Although the IgG4 level was normal and IgG4-bearing cells were sparse, we strongly suspected that the patient had IgG4-related disease, due to the appearance and distribution of the lesions. We reevaluated the preserved lymph node biopsy that was acquired in 1994 and the serum that was acquired in 1995. The lymph node showed lymphoid hyperplasia with lymphocytes and plasma cells. Immunohistochemical staining revealed that over half the plasma cells were positive for IgG4 (Figures 2(c), and 2(d)). Moreover, the serum IgG4 was high (317 mg/dL). Taking these findings together, we diagnosed that the patient had had IgG4-related disease from 1994, and that the current complaint was due to a relapse. The patient was given 50 mg (1 mg/kg) PSL daily, and the visual field abnormality and lymph node swelling improved rapidly. After 4 months of treatment, serum IgG levels declined to within the normal range and the abnormal ^67^Ga accumulation had disappeared. In October 2011, he was taking 5 mg PSL daily, and he has shown no signs of relapse.

The article "IgG4-Related Disease without Overexpression of IgG4: Pathogenesis Implications" was published in 2012. Journal: Case Rep Rheumatol.

## 3. Discussion

IgG4-related disease is a recently identified lymphoproliferative disorder characterized by hyper-IgG4-*γ*-globulinemia and IgG4-bearing plasma cell expansion in affected organs with fibrotic or sclerotic changes [5]. The disease frequently progresses in a variable pattern to involve one or multiple characteristic organs; however, the cause of this disease remains poorly understood.

In MRIs, IgG4-related disease can be characterized by hypophysitis in pituitary gland lesions [7], lymphadenopathy in the lymph node [8], inflammatory pseudotumors in the lungs [9], and multiple nodules in the kidney that lack contrast enhancement [10]. Two pathologic features characterize IgG4-related disease. First, hematoxylin and eosin staining shows lymphoplasmacytic infiltration, irregular fibrosis, occasional eosinophilic infiltration, and obliterative vasculitis, regardless of the affected organ [2]. Second, immunostaining shows a greater than 30% proportion of IgG4-positive to IgG-positive plasma cells [2]. In this study, at the current admission, the patient showed normal serum IgG4 concentrations and scarce IgG4-bearing cells in the affected tissues. However, taken together with the CT and MRI images, histopathological features of lymph nodes acquired at the onset showed greater than 50% infiltrations of IgG4-bearing plasma cells, which was consistent with a diagnosis of IgG4-related disease. Moreover, the serum from 15 years ago revealed high IgG4 levels (317 mg/dL). This led us to diagnose this case as IgG4-related disease, according to the criteria proposed by Masaki et al. as follows: (1) Characteristic diffuse/localized swelling or masses in single or multiple organs. (2) Serum IgG4 > 135 mg/dL. (3) Histopathological features that included lymphocyte and IgG4+ plasma cell infiltration (i.e., the proportion of IgG4+ plasma cells to IgG+ plasma cells > 40% and >10 IgG4+plasma cells/HPF), with typical tissue fibrosis [11].

The article "IgG4-Related Disease without Overexpression of IgG4: Pathogenesis Implications" was published in 2012. Journal: Case Rep Rheumatol.

Although the role of IgG4 in IgG4-related disease remains unknown, IgG4 has become a definitive marker; thus, we could discriminate IgG4-related disease from other inflammatory pseudotumors. In this regard, autoimmune pancreatitis is now classified into two distinct subsets, (type 1 and type 2), according to the presence or absence of infiltrating IgG4-positive plasma cells [12, 13]. However, interestingly, in this case, IgG4-positive plasma cells were abundant at the time of onset, but scarce at the time of relapse. It is unclear why IgG4-bearing plasma cell infiltration was scarce at the time of relapse; it may have been the result of long-term PSL treatment. However, the PSL dose was only 2 mg/day for over two years; this is likely to be too insubstantial to abolish infiltration.

 When patients diagnosed with IgG4-related disease are admitted during a relapse, a reevaluation of the histology tends to be omitted when the clinical presentation is typical of IgG4-related disease. The present study indicated that histological evaluations of specimens should be obtained from affected organs during the course of the IgG4-related disease; these specimens may provide important information on the pathogenesis of IgG4-related disease.

## Figures and Tables

**Figure 1:** Lesions in a patient with IgG4-related disease. (a) Head MRI on a T2-weighted image, sagittal section. A pituitary mass of 30 mm was detected (arrow). (b) Chest CT shows a nodule in the right lung (arrow). (c) Abdominal CT shows that part of the left kidney was not enhanced with contrast media (arrow). (d) ^67^Gallium accumulated abnormally in the pituitary gland, both sides of the neck, both lungs, both kidneys, and the left inguinal area (arrows).

**Figure 2:** Histopathology of the pituitary gland and lymph node in a patient with IgG4-related disease. (a) Hematoxylin and eosin staining of the pituitary gland (2010). Bar 100 *μ*m. The gland structure was unclear, and numerous lymphocytes and plasma cells had infiltrated the fibrous tissue. (b) Immunohistochemical staining of the pituitary gland for IgG4 showed that IgG4-positive cells were sparse; they comprised about 10% of all IgG-positive cells. Bar 200 *μ*m. (c) Hematoxylin and eosin staining of the lymph node (1994). Bar 100 *μ*m. Plasma cell infiltration was abundant. (d) Immunohistochemical staining of the lymph node for IgG4 showed abundant IgG4-bearing plasma cells; they comprised over 50% of all IgG-positive cells. Bar 200 *μ*m.
